# NR2F1-AS1 Acts as an Oncogene in Breast Cancer by Competitively Binding with miR-641

**DOI:** 10.1155/2022/6778199

**Published:** 2022-01-17

**Authors:** Yan Zhong, Weiwei Zeng

**Affiliations:** ^1^Department of Breast and Thyroid Surgery, Shenzhen Baoan Women's and Children's Hospital, Shenzhen 518102, China; ^2^Department of Pharmacy, Shenzhen Baoan Women's and Children's Hospital, Shenzhen 518102, China

## Abstract

**Background:**

Long noncoding RNA (lncRNA) NR2F1-AS1 has been previously reported to be dysregulated in human cancers and implicated in the tumorigenesis and development of tumors. In this research, we detected the expression level and biological function of NR2F1-AS1 in breast cancer (BC).

**Methods:**

The expression of NR2F1-AS1 in BC tissues and cell lines was determined by qRT-PCR analysis. The associations of NR2F1-AS1 expression with clinical characteristics and survival rate of BC patients were also analyzed. Cell proliferation, migration, and invasion were measured by the CCK-8 and Transwell assay.

**Results:**

The results revealed that the total survival time of BC patients with high NR2F1-AS1 expression was lower than that of BC patients with low NR2F1-AS1 expression. Moreover, functional experiments demonstrated that knockdown of NR2F1-AS1 inhibited BC cell viability, migration, and invasion abilities, whereas overexpression of NR2F1-AS1 had the opposite effect. Mechanistic investigation revealed that NR2F1-AS1 can competitively bind with microRNA-641 (miR-641) in BC. These results revealed that NR2F1-AS1 functioned as an oncogene by sponging miR-641 expression in BC cell progression. Moreover, miR-641 was negatively correlated with NR2F1-AS1 in BC tissues.

**Conclusion:**

Hence, NR2F1-AS1 was found to act as an oncogene in breast cancer by suppressing miR-641. We suggested that NR2F1-AS1 could be a potential biomarker for BC diagnosis and therapy.

## 1. Introduction

Breast cancer (BC) is reported to rank second in cancer incidence and fifth in cancer mortality [1]. In most countries around the world, the incidence and mortality of BC ranks first among women [2]. The World Health Organization estimates that about 1.3 million women are newly diagnosed with BC each year [3]. The incidence of BC among women in most countries and regions around the world is still rising [4]. Therefore, it is of great significance to study the pathogenesis and development mechanism of BC.

Long noncoding RNAs (lncRNAs) are a group of non-protein-coding transcripts. 16,000 lncRNAs have been identified in humans, but the vast majority of their functions are still unknown. Accumulating reports have discovered that numerous lncRNAs are implicated in a wide spectrum of biological processes of human diseases, such as X-chromosome silencing, tumorigenesis, cell proliferation, metastasis, prognosis, angiogenesis, and signaling pathways [5, 6]. In recent years, various lncRNAs have been reported to express abnormally and be involved in the tumorigenesis and progression of BC. For instance, DSCAM-AS1 was found to facilitate the tamoxifen resistance of BC and promote BC cell propagation by sponging miR-137 and upregulating EPS8 expression [7]. LINC00963 was demonstrated to be upregulated in BC tissues, and overexpression of LINC00963 promoted cell proliferation, tumorigenesis, and radioresistance through antagonization of miR-324-3p and regulation of ACK1 [8]. Inversely, Zhou et al. discovered that LET overexpression restrained cell proliferation, migration, and invasion in BC [9]. Moreover, WT1-AS was found to be a potential tumor inhibitor in triple-negative breast cancer [10]. NR2F1 antisense RNA 1 (NR2F1-AS1) has been reported to be pivotal in the tumorigenesis and development of human cancers. For instance, NR2F1-AS1 was markedly highly expressed in esophageal squamous cell carcinoma cells and droved cell proliferation by activating the Hedgehog signaling pathway [11]. Furthermore, Huang et al. revealed that NR2F1-AS1 silencing suppressed cell migration, invasion, and oxaliplatin resistance by regulating the miR-363/ABCC1 axis in hepatocellular carcinoma [12]. Nevertheless, the function of NR2F1-AS1 in BC is not fully understood.

MicroRNAs (miRNAs) are widely involved in various aspects of human physiology and pathology, including cell proliferation, apoptosis, differentiation, metabolism, hematopoiesis, virus defense, and tumor metastasis [13]. It is still a research hotspot to study the relationship between tumors and miRNAs. miRNA mutations, deletions, and changes in the expression play a role similar to proto-oncogenes or tumor suppressor genes in human tumors. miR-641 was found to act as a tumor inhibitor in lung cancer by inhibiting MDM2 expression and enhancing p53 expression [14]. Moreover, Yan et al. verified that miR-641 is regulated by targeting CYP3A4 in HepaRG cells [15]. However, the effect of miR-641 on the development of BC remains unclear.

In this article, we designed to measure the expression pattern of NR2F1-AS1 and miR-641 in BC tissues and BC cells. Moreover, the functions of NR2F1-AS1 and miR-641 on cell growth and metastasis in BC have also been explored in our research.

## 2. Materials and Methods

### 2.1. Clinical Information

54 BC tissues and adjacent tissues were obtained from Shenzhen Baoan Women's and Children's Hospital. All patients were diagnosed pathologically and had not received radiochemotherapy before surgery. After surgery, BC tissues and 2 cm tumor adjacent tissues were taken in liquid nitrogen immediately and then stored in a −80°C refrigerator. All patients or their families have written the informed consent. The experiments were approved by the Ethics Committee of Shenzhen Baoan Women's and Children's Hospital.

### 2.2. Cell Culture and Cell Transfection

Six human BC cell lines (MCF-7, MDA-MB-231, BT-474, MDA-MB-468, BT-549, and HCC1937) were purchased from the Type Culture Collection of the Chinese Academy of Sciences (Shanghai, China). The normal BC cell line (MCF-10A) was obtained from BeNa Culture Collection (Beijing, China). All BC cells were cultured in Dulbecco's modified Eagle's medium (DMEM, Gibco, USA) with 10% foetal bovine serum (FBS, Gibco, USA), 100 *μ*g/ml streptomycin, and 100 U/ml penicillin (Jinpin Chemical Technology Co., Ltd, China) at 37°C and 5% CO_2_. Then, 0.25% trypsin was used to passage cells every other day.

Specific small interference RNAs of NR2F1-AS1 (si-NR2F1-AS1), small interference RNAs of miR-641 (miR-641 inhibitor), pcDNA3.1-NR2F1-AS1 (NR2F1-AS1 vector), pcDNA3.1-miR-641 (miR-641 mimic), and their corresponding negative control (NC) were synthesized by GenePharma. Cells (2 х 10^5^ cells/mL) were inoculated into 6-well plates at 37°C and 5% CO_2_. We transfected those fragments into MCF-7 cells by using Lipofectamine 2000 (Invitrogen, Waltham, MA, USA).

### 2.3. RNA Extraction and Quantitative PCR Analysis

RNA samples were isolated from BC tissues and cells by using TRIzol reagent (Invitrogen, Carlsbad, CA). Then, the RNAs were reverse-transcribed into complementary according to the PrimeScript RT reagent kit (Invitrogen, Shanghai, China). Bio-Rad CFX96 and SYBR Green Premix Ex Taq II (Takara, Dalian, China) were used for qRT-PCR. LightCycler 96 thermocycler was used to investigate the relative expression of NR2F1-AS1 and miR-641. The expression of NR2F1-AS1 was normalized to GAPDH, while that of miR-641 was standardized to U6. The primer sequences were listed as follows: NR2F1-AS1, forward: 5′-CGCGAGGGCGTAAAAGTTTG-3′ and reverse: 5′-AGCGTGGCCATTTACTTCCA-3′; miR-641, forward: 5′-GGCTGGGTGAAAGGAAGGAA-3′ and reverse: 5′-GAGGCTCAGGGGTAAGAGGA-3′; GAPDH, forward: 5′-CCTGACCTGCGTGTGGACT-3′ and reverse: 5′-GCTGTGGATGGGGAGGTGTC-3′; and U6, forward: 5′-CTCGCTTCGGCAGCACA-3′ and reverse: 5′-TGGTGTCGTGGAGTCG-3′.

### 2.4. Dual-Luciferase Reporter Assay

NR2F1-AS1-mut or NR2F1-AS1-wt and miR-641 mimic or miR-NC were transfected into MCF-7 cells by Lipofectamine 2000 (Invitrogen, Waltham, MA, USA). MCF-7 cells were cultured at 37°C, 5% CO_2_, and 95% humidity. After incubation for 48 hours, the luciferase activity of NR2F1-AS1 was estimated by the dual-luciferase reporter assay system (Promega, USA).

### 2.5. CCK-8 Assay

The CCK-8 assay was adopted to assess the cell viability of BC cells. MCF-7 cells (1 × 10^3^ cells/mL) transfected with NR2F1-AS1 or miR-641 mimic were cultured into 96-well plates. After incubation in the incubator (37°C and 5% CO_2_) for 24, 48, 72, and 96 hours, CCK-8 solution (10 *μ*l) was added to each well. Incubation was continued in the incubator for 2 hours, and then the absorbance was measured with a microplate reader at 450 nm.

### 2.6. Transwell Assay

Transwell chambers (8 *μ*m; Millipore) were used to examine BC cell migration and invasion abilities. Cell migration was detected without Matrigel, whereas cell invasion was detected in the upper chamber with Matrigel. First, cells (1 × 10^3^ cells/mL) were inoculated in the upper Transwell compartment. Then, 10% FBS was added into the lower compartment. After being cultivated at 37°C for 24 h, the cells were fixed and stained with 0.5% crystal violet. Finally, the invasive and migratory cells were counted under an optical microscope.

### 2.7. Statistical Analysis

The experimental results were analyzed by using GraphPad Prism 6.0 and SPSS 20.0. Also, data were presented as mean ± standard deviation. The comparison between multiple groups was analyzed by one-way ANOVA followed by Tukey's post hoc test. The pairwise comparison was performed by Student's *t*-test. The correlation between NR2F1-AS1 and miR-641 in BC tissues was measured by Pearson's correlation analysis. *p* < 0.05 is considered statistically significant.

## 3. Results

### 3.1. NR2F1-AS1 Expressed at a High Level in BC Tissues and Cells

To explore the expression mode of NR2F1-AS1 in BC, we primarily detected the expression level of NR2F1-AS1 in 54 BC tissues. RT-qPCR results displayed that NR2F1-AS1 was highly expressed in BC tissues than in normal tissues (Figure 1(a)). Similarly, NR2F1-AS1 was upregulated in BC cell lines (MCF-7, MDA-MB-231, BT-474, MDA-MB-468, BT-549, and HCC1937) compared with MCF-10A cells (Figure 1(b)). Based on the average expression value of NR2F1-AS1, we divided 54 BC patients into the high expression group and low expression group. The correlation between NR2F1-AS1 expression and clinical characteristics of 54 BC patients was analyzed by the chi-squared test. As presented in Table 1, the overexpression of NR2F1-AS1 was closely related to the TNM stage and lymph node metastasis. Furthermore, the high NR2F1-AS1 expression group had shorter overall survival (OS) time than the low group (Figure 1(c)). These results revealed that NR2F1-AS1 was upregulated in BC and associated with poor prognosis of BC patients.

### 3.2. Depletion of NR2F1-AS1 Repressed Cell Proliferation, Migration, and Invasion in BC

Based on the abovementioned experimental results, MCF-7 cells were selected for the functional experiments. To measure the function of NR2F1-AS1 in BC, NR2F1-AS1 si-RNA was transfected into MCF-7 cells. The data showed that the expression level of NR2F1-AS1 was obviously declined by si-NR2F1-AS1 transfection (Figure 2(a)). Next, cell proliferation was explored by the CCK-8 assay. The Transwell assay was used to assess BC cell migration and invasion ability. As shown in Figure 2(b), depletion of NR2F1-AS1 weakened cell proliferation ability in MCF-7 cells. Moreover, the number of migrated and invaded cells was reduced by NR2F1-AS1-silencing transfection (Figures 2(c) and 2(d)). Our data verified that depletion of NR2F1-AS1 repressed cell progression in BC.

### 3.3. Upregulation of NR2F1-AS1 Promoted Cell Proliferation, Migration, and Invasion in BC

Furthermore, we measured the function of upregulation of NR2F1-AS1 on cell proliferation, migration, and invasion in MCF-7 cells. The results showed that the NR2F1-AS1 vector notably increased the expression level of NR2F1-AS1 (Figure 3(a)). Functionally, we noticed that MCF-7 cell proliferation was accelerated by the NR2F1-AS1 vector (Figure 3(b)). Similarly, the NR2F1-AS1 vector significantly increased the number of migrated and invasive cells of MCF-7 cells (Figures 3(c) and 3(d)). Previous results demonstrated that NR2F1-AS1 acted as a carcinogen in the progression of BC.

### 3.4. NR2F1-AS1 Can Function as a Sponge of miR-641 in BC

lncRNAs were found to act as ceRNAs of various miRNAs in human cancers. In this study, the Starbase software predicted that there were special binding sites between NR2F1-AS1 and miR-641 (Figure 4(a)). To verify this prediction, the dual-luciferase reporter assay was adopted to detect the luciferase activity of NR2F1-AS1-mut and NR2F1-AS1-wt. We observed that miR-641 mimic declined the luciferase activity of NR2F1-AS1-mut but had no influence on NR2F1-AS1-wt (Figure 4(b)). To explore the relationship between NF2F1-AS1 and miR-641, the RT-qPCR assay was adopted to measure their expression levels. We found that the expression of miR-641 was decreased by the NR2F1-AS1 vector but increased by si-NR2F1-AS1 (Figure 4(c)). Moreover, miR-641 mimic decreased the expression of NR2F1-AS1, whereas miR-641 inhibitor increased the expression of NR2F1-AS1 (Figure 4(d)). As a consequence, we suggested that NR2F1-AS1 can be a sponge to regulate miR-641 expression in BC.

### 3.5. NR2F1-AS1 Regulated BC Cell Progression by Modulating miR-641 Expression

Next, we assessed the expression level of miR-641 in BC tissues. As presented in Figure 5(a), there was a downexpression of miR-641 in 54 BC tissues. Moreover, miR-641 was lowly expressed in BC cell lines than in normal cell line (Figure 5(b)). Moreover, to investigate the function of NR2F1-AS1/miR-641 on the progression of BC, the NR2F1-AS1 vector was transfected into MCF-7 cells with miR-641 mimic. RT-qPCR results indicated that miR-641 expression was elevated by miR-641 mimic, while decreased by the NR2F1-AS1 vector transfected into miR-641 mimic (Figure 5(c)). Functional experiments displayed that miR-641 mimic retarded cell proliferation of MCF-7 cells, while NR2F1-AS1 upregulation weakened the suppression effect of miR-641 mimic (Figure 5(d)). Furthermore, miR-641 overexpression suppressed cell migration and invasion ability of MCF-7 cells, while the NR2F1-AS1 vector increased the number of migrated and invasive cells of MCF-7 cells (Figures 5(e) and 5(f)). Furthermore, Pearson's correlation analysis indicated that NR2F1-AS1 negatively correlated with miR-641 in BC tissues (Figure 5(g)). All data demonstrated that NR2F1-AS1 accelerated the BC cell proliferation and metastasis by counteracting miR-641 expression.

## 4. Discussion

Recent experiments have shown that lncRNAs are expected to become new biomarkers for the clinical diagnosis and treatment of human tumors [16]. In this research, we found an increased expression of NR2F1-AS1 in 54 BC tissues and 6 BC cell lines. Consistent with our findings, NR2F1-AS1 was reported to be upregulated in papillary thyroid carcinoma [17] and neuroblastoma [18]. Functionally, we noticed that depletion of NR2F1-AS1 retarded cell growth, migration, and invasion of BC cells. In addition, the overexpression of NR2F1-AS1 promoted the cell viability of BC cells. Consistent with our findings, in endometrial cancer, NR2F1-AS1 inhibition prevented cell viability, migration, and invasion by interplay with miR-363/SOX4 [19]. Furthermore, Guo et al. discovered that NR2F1-AS1 enhanced cell growth and restrained cell apoptosis by modulating miR-338-3p and CCND1 in thyroid cancer [20]. Different from previous studies, NR2F1-AS1 was lowly expressed in cervical squamous cell carcinoma cells, and upregulation of NR2F1-AS1 repressed cell metastasis viability by targeting miR-17 and upregulating SIK1 [21]. Furthermore, NR2F1-AS1 was found to be closely associated with the TNM stage and lymph node metastasis in BC. All findings indicated that NR2F1-AS1 functioned as a carcinogen in the development of BC, and NR2F1-AS1 was related to poor prognosis of BC patients, which was as same as Liao's study [22].

lncRNAs act as competitive endogenous RNAs (ceRNAs) of a large number of miRNAs in human tumors. In previous research studies, miR-34b-5p [23], miR-101 [24], and miR-638 [25] were found to act as a BC tumor suppressor, while miR-96-5 [26], miR-146 [27], and miR-15b [28] promoted BC progression. In osteosarcoma, NR2F1-AS1 was found to be competitively bound with miR-483-3p [29]. In our study, we verified that NR2F1-AS1 acted as a sponge of miR-641 in BC by using the Starbase software. Furthermore, miR-641 was discovered to be decreased in BC tissues and cell lines. Similarly, miR-641 was with a low expression level in gastric cancer [30]. Functionally, we noticed that miR-641 overexpression restrained cell proliferation, migration, and invasion in MCF-7 cells. Consistent with our results, miR-641 retarded cell viability and metastasis in non-small-cell lung cancer [31] and osteosarcoma [32]. Unlike previous findings, an increased expression of miR-641 was discovered in cervical cancer, and miR-641 inhibitor reduced cell migration and invasion capacity [33]. Furthermore, the NR2F1-AS1 vector neutralized the inhibition effect induced by miR-641 overexpression. Simultaneously, we verified that there was an opposite correlation between NR2F1-AS1 and miR-641. Hence, our findings indicated that NR2F1-AS1 regulated BC cell progression and metastasis by competitively binding with miR-641.

## 5. Conclusion

In conclusion, our study reveals that NR2F1-AS1 is upregulated in BC and demonstrates the function of NR2F1-AS1 in promoting cell growth and metastasis capability of BC cells. In addition, we find that NR2F1-AS1 acts as a sponge of miR-641 in BC. Our research suggests that NR2F1-AS1 can function as a biomarker for BC diagnosis and treatment.

## Figures and Tables

**Figure 1:** NR2F1-AS1 was expressed at a high level in BC tissues and cell lines. (a) The expression of NR2F1-AS1 in BC tissues and adjacent normal tissues. (b) The relative expression of NR2F1-AS1 in BC cell lines. (c) The survival rate for low NR2F1-AS1 expression and high NR2F1-AS1 expression. ^*∗∗*^*p* < 0.01.

**Figure 2:** Depletion of NR2F1-AS1 retarded cell proliferation, migration, and invasion in BC. (a) The relative expression of NR2F1-AS1 in MCF-7 cells with si-NR2F1-AS1. (b) The cell proliferation ability of MCF-7 cells with si-NR2F1-AS1. (c, d) The cell migration and invasion of MCF-7 cells with si-NR2F1-AS1 (scale bar = 100 *μ*m). ^*∗∗*^*p* < 0.01.

**Figure 3:** Upregulation of NR2F1-AS1 promoted cell proliferation, migration, and invasion in BC. (a) The relative expression of NR2F1-AS1 in MCF-7 cells with the NR2F1-AS1 vector. (b) The cell proliferation ability of MCF-7 cells with the NR2F1-AS1 vector. (c, d) The cell migration and invasion of MCF-7 cells with the NR2F1-AS1 vector (scale bar = 100 *μ*m). ^*∗*^*p* < 0.05; ^*∗∗*^*p* < 0.01.

**Figure 4:** NR2F1-AS1 can function as a sponge of miR-641 in BC. (a) The binding sites between NR2F1-AS1 and miR-641. (b) The relative luciferase activity of NR2FA-AS1-wt and NR2F1-AS1-mut. (c) The relative expression of miR-641 in MCF-7 cells with si-NR2F1-AS1 or NR2F1-AS1 vector. (d) The relative expression of NR2F1-AS1 in MCF-7 cells with miR-641 inhibitor or miR-641 mimic. ^*∗∗*^*p* < 0.01.

**Figure 5:** NR2F1-AS1 regulated cell progression by modulating miR-641 expression in BC. (a) The relative expression of miR-641 in BC tissues. (b) The relative expression of miR-641 in BC cell lines. (c) The relative expression of miR-641 in MCF-7 cells transfected with the NR2F1-AS1 vector and miR-641 mimic. (d) The cell proliferation in MCF-7 cells transfected with the NR2F1-AS1 vector and miR-641 mimic. (e, f) The cell migration and invasion ability in MCF-7 cells transfected with the NR2F1-AS1 vector and miR-641 mimic. (g) NR2F1-AS1 had a negative correlation with miR-641 in BC tissues. ^*∗∗*^*p* < 0.01; ^##^*p* < 0.01.

**Table 1:** Correlation between the expression level of NR2F1-AS1 and clinical characteristics of BC patients (*n* = 54).

Clinical characteristics	Number of cases (*n* = 54)	NR2F1-AS1 expression	
		Low (*n* = 25)	High (*n* = 29)	*p* value
Age (years)				0.510
≥50	32	16	16	
<50	22	9	13	
Tumor size				0.300
≥2 cm	24	13	11	
<2 cm	30	12	18	
Lymph node metastasis				0.003^*∗∗*^
Absent	36	22	14	
Present	18	3	15	
ER status				0.419
Negative	26	12	14	
Positive	28	16	12	
TNM stage				0.028^*∗*^
I-II	42	23	21	
III	12	2	10	

^*∗*^ *p* < 0.05, the difference is significant; ^*∗∗*^*p* < 0.01, the difference is highly significant.

## Data Availability

The datasets used and/or analyzed during the current study are available from the corresponding author on reasonable request.
